# Global Value Chain Governance of the Apparel Design Industry under the Background of Global Sustainable Economic Development

**DOI:** 10.1155/2022/5178301

**Published:** 2022-12-02

**Authors:** Dan Yu, Peipei Zhao

**Affiliations:** Department of Fashion Design, Academy of Fine Arts and Design, Changchun Humanities and Sciences College, Changchun 130000, China

## Abstract

In recent years, there has been a significant rise in the importance of sustainability in business and personal life. Unsustainable techniques are used throughout the whole lifecycle of the clothing and textiles business, from the time it is made to the time it is recycled or thrown away. The garment sector and its customers must be ready for a more sustainable future as the government, corporations, and society turn their focus toward it. An investigation of how the apparel design industry (ADI) might adhere to the global value chain (GVC) in light of sustainable economic development (SED) and their relevance in China. This study analyzes the ADI moves up from one functional level to another within the global apparel value chain and what factors allow them to break into the global market. Researchers demonstrate that the existing sustainable operations in the AD industry are a long way from attaining the aims of economic development going hand in hand with the goals of economic sustainability by studying both the relevant literature and the industrial practices in the sector. This study relies on various case studies, proposes the “apparel global value chain” of governance-based sustainability, explores the implications of these models for areas with very varied degrees of development and diverse AD structures, and considers their implications for regional development and sustainability. As a development of a better knowledge of how fashion design contributes to economic sustainability. The study aims to examine how ADI uses economically sustainable techniques and how designers contribute to the creation of environmentally friendly goods.

## 1. Introduction

Sustainable economic development (SED) is an excellent illustration of the new goals of economic, social, and environmental development. These new goals include things like eradicating poverty, fostering economic growth, and protecting the environment, among other things. SED needs participation from all global actors including governments, businesses, nonprofits, and individuals in order to achieve their objectives are stated by Jia et al. [1]. An export-oriented strategy of industrialization and China's membership in global value chains (GVCs) and global production networks (GPNs) have contributed, at least in part, to the phenomenal economic development that China has seen in recent decades. China's gradual transition towards a marketized, globalized, and privatized economy over the past few decades has generated dramatic economic growth, with an average annual GDP growth rate of 9.8 percent and its exports increasing by 10–20 percent annually. This has resulted in a dramatic increase in China's overall standard of living. However, hiding beneath China's recent economic success is the country's huge dependency on low-wage labor that is untrained or semiskilled, as well as its heavy use of home advantages to its benefit. This low-wage export-oriented expansion has been illustrated by the garment sector, which has been responsible for a significant portion of China's economic growth as well as the creation of new jobs. When compared to supply chains in other industries, the fashion supply chain is notable for its labor-intensive manufacturing, lengthy value chain, and relatively high level of environmental pollution. The encouraging growth of China's export-oriented apparel firms can be attributed, in large part, to the following factors: (1) the flexible business environment, which includes cheap peasant workers who migrate from the western and central regions to coastal China, and China's other low-cost factor inputs, land electricity, and raw materials; (2) lax inspection on import materials and export products in customs; (3) halfhearted implementation of environmental and labor regulations; and (4) preferential Taiwanese trade agreements. According to Gazzola et al. [2] mentioned that the fashion supply chain is part of the global value chain that is associated with the textile and apparel industry.  Figure 1 depicts the sustainable growth in each country. Although it is the second biggest exporter of garments, Bangladesh has yet to establish itself as a leading textile production and exporting nation. China continues to dominate the global textile market, followed by the EU, India, Turkey, Vietnam, and Hong Kong, respectively. In order for Bangladesh to achieve long-term success in the clothing sector, it is necessary for the country to expand its textile production capabilities. This will ensure that the country's clothing exports are no longer reliant on foreign textile imports.

The global production system capitalizes on the relatively cheap cost of labor in emerging nations from both an economic and a social point of view.  Figure 2 indicates the principles of achieving sustainability. The manufacturing of garments is one of the engineering processes with the highest risk. The wet processing sector in particular generates a significant quantity of effluents, which significantly contribute to the pollution of our water base. Therefore, in order to achieve sustainable growth in the textile industries, it is necessary to take into account the industries' potentially harmful effects on the surrounding environment and to put in place appropriate mitigation strategies. These four principles should be adopted by the industry if it is to have any hope of achieving sustainable development. However, there are fees associated with accomplishing all of these goals. When it comes to business, adhering to sustainable ideals cannot come at the expense of competitiveness. That is the balance that the sector has to figure out in order to adopt sustainable practices in a gradual manner so that the extra expenses connected with becoming sustainable do not influence the competitiveness of the company.

Major goals for economic growth in low-income countries (LICs) continue to be structural change and export diversification away from basic commodities and towards items with greater value-added LICs. The apparel industry has historically been a gateway for LICs to diversify their exports, and it is generally regarded as the first step for developing countries that are beginning the process of export-oriented industrialization. Historically, the apparel industry has been a gateway to export diversification. As a result of its low entry hurdles (low fixed costs and relatively basic technology), the apparel industry was able to hire vast numbers of unskilled employees are reported by Nguyen et al. [3] and Moretto et al. [4]. In turn, this opened up prospects for upgrading into activities with better value-added both inside and across industries. However, the features that define this industry also imply that it is very competitive. As a result, many suppliers have little leverage, and it might be difficult to ensure that longer-term development gains will be realized. This research examines how the ADI climbs through the global clothing value chain from one functional level to the next, and what criteria enable them to break into the global market. The “apparel global value chain” of governance-based sustainability is proposed, and the consequences of these models for regions with widely varying degrees of development and widely varying AD structures are explored and considered in this paper, which is based on several case studies.

### 1.1. Contributions of this Research

- For the evaluated apparel global value chain, the apparel industry has a special position in the sustainable economy. The country's most significant industry is this one, which makes up the bulk of exports overall and has had tremendous growth over the last 20 years.
- The economy has a critical role in both the process of generating employment and the transfer of funds to those who are less fortunate.
- Establishing a cost-cutting strategy and a labor productivity cell to conduct a range of research in this field, as well as other supporting policies important to the growth, development, and survival of the apparel industry in the many countries under consideration SED.

These may be helpful in addressing the issues, and value addition will enable the garment industry's contribution to the socioeconomic development of nations to be strengthened and sustained through time.

The additional detail of this survey is as follows: Section 2 briefly presents the global organization of the apparel design industry.  Section 3 explains the apparel global value chain. In Section 4, the economic improvements in the global apparel value chain are mentioned.  Section 5 discusses the apparel global value chain contextualization and sustainable development.  Section 6 discusses the relationship between apparel value chains and SEDs.  Section 7 described the discussion and analysis of the country cases.  Section 8 explains the conclusion of this survey.

## 2. Global Organization of the Apparel Design Industry

The apparel industry is the perfect illustration of a buyer-driven commodity chain, since it is characterized by power imbalances between the worldwide consumers of finished fashion goods and the providers of those products are asserted by Gardas et al. [5]. The most economical products may be found in these companies. Lead businesses often have their headquarters in the main markets, which include Europe, Japan, and the United States. These firms include merchants, as well as owners of brand names, are suggested by Nayak et al. [6]. In the apparel value chain, these organizations are frequently responsible for the most critical activities such as industrial design, advertising, and sales, and they subcontract the manufacturing process to a global wide range of suppliers (Goworek et al. [7]).  Table 1 indicates the employment in the apparel industry in a few countries.

The value chain of the garment industry, like the value chains of other global businesses, depends on international standards to coordinate the operations of its suppliers. By the turn of the century, the majority of leading companies had already developed their own internal standards and codes of conduct based on factors such as cost, quality, punctuality, and corporate responsibility in terms of labor and environmental norms (Hur and Cassidy [8] and Mody and Bhoosreddy [9]). Regular measurements are taken to assess the functioning of the factory, and delivery, quality, and pricing are monitored throughout time. It is not uncommon for businesses to have certifications from a number of different companies are indicated by Pedersen et al. [10].

## 3. Apparel Global Value Chain

One of the most important parts of the apparel value chain is the resource of organic and inorganic fiber natural resources; the manufacturing of garment elements; the output networks founded by barter proxies; the advertising systems at the retail stage; and the availability of raw materials of apparel global value chain as shown in Figure 3. There has been consistent movement throughout the course of history in the locations of the most important nations and areas for the export of garments, as well as the primary end markets for those exports (McEachern et al. [11] and Choi and Luo [12]).

The worldwide value chain in the apparel sector is a great illustration of a “buyer-driven” business model. A buyer-driven global garment value chain generates profits via a variety of high research, development, selling, advertising, and financial sectors, as opposed to manufacturer chains wherein revenues are earned through increasing size, quantity, and technical advances. In this way, they may serve as strategic intermediaries between manufacturers, distributors, and retailers throughout the world and the product niches they serve in their primary markets at residence (Khan et al. [13]). Anner [14] estimated that companies effectively control how fundamental value-adding activities are distributed along the value chain.

It is possible to identify six key value-adding activities, which will help you understand how this division of labor happens and how attempts to improve the workforce may alter the role emerging nations play in the global value chain (Frederick et al. [15] and Staritz and Whitfield [16]). (1) *R* & *D*, (2) design, (3) purchasing, (4) logistics (buying and distribution), (5) marketing and branding, and (6) services are the six pillars of an organization's apparel global value chain's curve of value-added stages are seen in Figure 4. Because the most significant value-adding stages are intangible services that take place before and after the process of producing apparel, this model requires us to significantly expand our ideas regarding the locations that are most likely to experience the greatest benefits as a result of workforce development are reported by Prabowo et al. [17].

The most important value-adding stages include the following:

- *R* & *D*: companies that participate in research and development (*R* & *D*) as well as actions aimed at enhancing the physical product or process, as well as market and consumer research, falls within the purview of this value-adding function.
- Design: at this point in the value chain, a variety of persons and businesses are involved in providing services related to the esthetic design of various goods and components. Activities related to design and style are used to draw attention, enhance product performance, reduce manufacturing costs, and provide the product with a significant competitive edge in the market that is being targeted.
- Purchasing: this stage relates to the procedures involved in acquiring and delivering apparel items, which are known as inbound processes. It encompasses not only the actual act of moving things, but also the management of, or provision of, the technology and equipment necessary for supply chain coordination. Coordination in logistics may take place either inside a country or outside.
- Production: fabric may be woven or knitted, and then either the fabric or the garment can be cut and sewn straight from the yarn. The cut-and-sew categorization refers to a wide variety of businesses that produce whole lines of ready-to-wear as well as bespoke clothing. The term “apparel manufacturer” may refer to either an independent contractor who carries out cutting or sewing operations on materials held by third parties or a jobber or tailor who creates customized clothing for particular customers. Companies have the option of acquiring textiles from another organization or producing the textile components themselves.
- Distribution: there are a large number of companies that help supply and sell the clothing once it has been manufactured. These include merchants and agents as well as transportation and logistics companies.
- Marketing: afterward, the apparel is disseminated and marketed via a network of distributors, brokers, and other companies that are responsible for value-added operations that are not directly related to the manufacturing system.
- Services: this encompasses any form of activity that a company or industry delivers to its suppliers, customers, or workers, generally as a strategy to differentiate itself from rivals in the market (for example, delivering consultancy services about international clothing enterprises or fashion trends) (Whitfield et al. [18]).

## 4. Economic Improvements in the Global Apparel Value Chain

The apparel industry's purchaser responsibilities and expectations updating prospects operational (crossing to higher-value functions), consumer (producing higher-value items), procedural (incorporating sophisticated technologies into production), and multisectoral (moving across companies) (Garg [19] and Casadei and Iammarino [20]).

The following descriptions of the four primary phases of economic upgrading for the apparel industry are seen in Figure 5. The functional upgrading that occurs in the garment value chain is as follows:

- Assembly/cut make and trim (CMT) entry into the chain: in this step of the clothing business, sewing factories assemble foreign inputs. The manufacturer cuts, sews, trims, and ships the finished garment. The customer buys fabric and gives it to the maker with production specs. The contract manufacturer has many clients and takes orders. “Export-Processing Zones (EPZs),” special in economic zones, exports to the buyer's nation are taxed less.
- “Free on board (FOB)/full package/original equipment manufacturing (OEM)”: the garment maker handles CMT, finishing, and distribution. The company must be able to procure and finance raw materials, component items, and trim. According to Uramoto et al. [21] the circumstances, the buyer specifies textile businesses from which the apparel maker must acquire materials. In other cases, the company must build its own network of suppliers. The company frequently handles downstream logistics, including packing for retail distribution and transporting the finished product to the customer at an agreed fee (also referred to as FOB). The customer gives the FOB contractor product specs and designs but isn't engaged in pattern creation. Full-service enterprises might be single-producing operations or global suppliers with many production sites and product lines. Full package enterprises might source foreign or domestic fabrics. This method may generate major backward links to the textile industry, and many nations start textile production by making textiles for export are claimed by Ahmed et al. [22] and Rana et al. [23].
- “Original design manufacturing (ODM)/full package with design”: it combines design and production. Full-service garment suppliers design, purchase fabric, cut, sew, trim, package, and distribute completed garments (Wilson [24]). Typically, the supplier organizes and coordinates product design, sample approval, material selection, buying, manufacturing, and delivery to the ultimate client. Private-label retail companies often have full packaging designs (Mohajeri et al. [25]).
- “Original brand manufacturing (OBM)”: this business strategy adds or replaces design and production with product branding; upgrading entails selling own-brand items. Many developing nations engage OBM to establish brands for home or nearby markets.

## 5. Apparel Global Value Chain Contextualization and Sustainable Development

In the garment industry, like in many other industries, manufacturing and commerce are organized into GVCs, which include the manufacture of components and the assembly of those components into finished goods via interfirm networks operating on a worldwide scale. According to Uduwela et al. [26] stated that the apparel business is characterized by decentralized, internationally scattered manufacturing networks. These networks are controlled by lead corporations that oversee “value-added” operations (such as design and branding), but they often outsource production to a worldwide network of suppliers (Athukorala and Ekanayake [27] and Roy et al. [28]). Although buyers are not directly engaged in the manufacturing process, they exert a large amount of influence over producers by providing comprehensive product and production requirements. Because of this, the techniques that purchasers use, particularly their policies towards global sourcing, significantly impact the patterns of production and trade. Given the labor-intensive nature of garment manufacture, choices about sourcing are driven by differences in the cost of labor in various locations. However, in addition to the traditional factors of cost, quality, and dependability, additional factors are playing an increasingly important role in the decision-making process regarding sourcing are stated by Corvellec and Stal [29]. First and foremost, there has been a rise in the need for flexibility, but at the same time, lead times have decreased (Jung et al. [30] and Wang et al. [31]). This calls for more efficient supply chains and manufacturing processes. In addition, there is a necessity for nonmanufacturing competencies, such as the sourcing of inputs and the creation of products. Shahabaz et al. [32] and Jha and Kumar [33] mentioned the administration of inventories and stock holding, the logistics of shipping, and the financing of operations. Lastly, there is the need to comply with established labor and environmental norms, which has evolved into a baseline requirement for both entry into and continued participation in value chains as mentioned by Gomes et al. [34]. A consolidation of the supply base has occurred as a result of the sourcing strategies of buyers, which has resulted in a reduction in the number of supplier nations and enterprises within those countries. Conforming to Ahmad and Kamruzzaman [35] the competent suppliers who are confronted with high expectations on price, quality, and lead time, as well as high and shifting volume needs, and requests for wider nonmanufacturing competencies, have also sought to position themselves as coordinators of networks with a worldwide supply base. As a result, big manufacturers, particularly those based in Hong Kong, South Korea, and Taiwan, have transitioned into the role of middlemen, organizing dispersed international production and sourcing networks. They have become a major source of foreign direct investment (FDI) in the clothing export sectors of LICs and give a chance for new supplier nations to join apparel global value chains despite the fact that they have poor capabilities. In accordance with Donmezer et al. [36], there is a triangular manufacturing network, and the barriers to the entrance are much lower, but upgrading prospects are also restricted since the intermediaries have influence over the most important choices and tasks. More lately, there have also been advancements that enhance the continued extension of the supply base (Choi and Shi [37] and Alam and Dhamija [38]). This is something that has been happening more often as of late. As a result of cost rises in key supplier nations in Asia, buyers have been looking for new options in order to diversify their exposure to risk.  Figure 6 illustrates the sustainable development of the apparel industry. Bangladesh's clothing exports are second behind China with a 6.5% market share. The graphic shows that the clothing business has significant development potential since China's deficit is large. The textile sector must develop to fulfill yarn and fabric demand.

As determined by Jin et al. [39] a direct consequence of this, buyers or key suppliers have been screening new supplier countries in the hopes of finding ones that can at least partially replace or lessen their dependency on Bangladesh, China, and other Asian nations. Since tariffs (and consequently preferential market access) continue to play an important part in global apparel trade, preferential market access has continued to play an important role in the search for new sourcing locations are claimed by Bizuneh and Tadesse [40] and Dunhaupt et al. [41]. This has been the case in the apparel industry as it has been in the past. In addition to bilateral and multilateral trade agreements, wealthy nations have also participated in the generalized system of performance (GSP), which has granted tariff preferences to more than one hundred developing countries. However, the usual GSP for both the EU and the US only provides a little reduction in tariffs for items related to the garment industry Prasad et al. [42] and Li [43]. However, some nations have successfully secured preferential access for the world's least developed countries (LDCs), such as the Everything But Arms (EBA) agreement that the European Union has in place. Other relevant accords include the EU's “Economic Partnership Agreements (EPAs)” and the US's “Africa Growth and Opportunity Act (AGOA).”

As a result, LDCs in sub-Saharan Africa have been subjected to zero tariffs in European Union markets for a considerable amount of time; nevertheless, this has been accompanied by double transformation rules of origin (ROO). As specified by Bernardi et al. [44] and Abdeen et al. [44]. Single transformation became the standard for EBA ROOs in 2011. The newly agreed interim EPAs include single transformation requirements as an additional requirement. On the other hand, the EU grants preferential market access to all LDCs, which means that countries like Bangladesh and Cambodia may also export duty-free goods to the EU are stated by Jacobs and Karpova [45]. Only in 2001 did AGOA become fully operational, and it was only recently extended until the year 2025. It provides duty-free access for garment exports under specific criteria, with less-developed nations suffering single transformation ROOs in accordance with the third-country fabric (TCF) exemption indicated by Akter et al. [46]. The fact that AGOA grants duty-free access to the US market in clothing to only SSA and regional supplier nations in Central America is one of the program's most significant benefits specified by Salihu et al. [47] and Wang et al. [48]. LDCs in Asia are subject to tariffs. The value of AGOA is increased for the SSA nations because they now have a competitive advantage over the Asian suppliers. This is not the case with the preferential market access offered by the EU. Because of the severe rivalry that exists in the global textile and apparel industry, suppliers must implement strategies of upgrading in order to maintain and strengthen their positions in value chains in order to be successful. The term “upgrading” refers to the process of shifting toward activities that have a greater value in order to maximize the advantages derived from participation in global production are determined by Mark–Herbert and Ng [49]. In order to accomplish this improvement, the following procedures have been presented as possible solutions:

- Upgrade of processes (the improvement of technologies or industrial systems in order to achieve efficiency and flexibility)
- Product upgrading (the transition to goods that are more complicated and sophisticated)
- Modernization of the supply chain (including the establishment of domestic links, most particularly reverse linkages to input industries)
- Upgrade of the end market (diversifying to new consumers or expanding into new geographic and product markets)
- Functional upgrading refers to extending the variety of functions that can be performed or shifting the balance of activities to include more high-value activities

Functional upgrading is important for garment providers, including a CMT manufacturer that sews, cuts, and trims clothing (buttons, zippers). Buyer supplies product specs and fabric. Instead of a product price, the manufacturer receives a processing charge. A full-package manufacturer FOB offers textile inputs, manufacturing, finishing, and packaging. The buyer selects textile suppliers. ODMs participate in product design and development, including sample approval and material selection, purchasing, and manufacturing are claimed by Vishwakarma et al. [50]. OBMs create and promote their own brands. Sustainable development requires upgrading to stay competitive in GVCs and ensure local advantages, such as learning, technology transfer, value addition, and employment. Low costs typically mean low salaries, bad working conditions, and inadequate social and environmental norms. As believed by Bang et al. [51], social and environmental upgrading is connected with economic upgrading. Social upgrading improves employees' working conditions and rights, enhancing their employment. Skill upgrading comprises capturing learning and transferring skills to local labor. Environmental upgrading involves safeguarding ecosystem assets (clean water and energy) and natural resources to improve production and infrastructure's environmental performance. A comprehensive upgrading plan aims to promote inclusion, good jobs, reduced environmental consequences, and economic advantages and competitiveness.

## 6. Relationship between Apparel Value Chains and the SEDs

The apparel industry has undergone significant economic upgrading processes (in terms of end market, process, product, and function). A value chain is a collection of operations that a corporation operating in a certain sector does in order to offer a useful product or service to the market. There are, concurrently, localization processes in terms of local linkages that go beyond the experience of the other main apparel exporting countries in sub-Saharan Africa (SSA) determined by Patti and Acierno [52]. This is true once more with the exception that these processes are just starting, and there are no conclusive outcomes that can be observed just yet. In terms of social upgrading, there are favorable results from the standpoint of quantity, with less progress being achieved in terms of quality. Significant actions are now being taken, notably in the areas designated as industrial parks, with regard to the preservation of the natural environment.

## 7. Discussion and Analysis of the Country Cases

The accessibility to end markets, the availability of inexpensive labor in abundance, and advantageous trade agreements are the key prerequisites for successful entrance. Although foreign direct investment is often helpful in developing assembly operations, 4 of the 5 nations surveyed joined the sector primarily due to advantageous trade agreements. Prior to Lesotho and Nicaragua benefiting from the African Development and Opportunity Act (AGOA) and CAFTA-DR TPL accords, respectively, Lesotho and Sri Lanka profited greatly from preferential trade deals with the EU and the United States, which aided their early admission and growth.

Other aspects, meanwhile, start to matter as the chain advances into more advanced phases. They consist of the following:

- Domestic or regional textile industry facilitates upgrading from assembly (CMT) to full-package (OEM) garment manufacture. Bangladesh's emerging textile sector helped it transition from assembly to full-package supply. Turkey's textile sector was robust when the clothing industry was founded, enabling it to jump into full-package supply. Sri Lanka used regional textile possibilities and backward links with India and Bangladesh to upgrade.
- Lead businesses' nationality and business methods determine a country's upgrading trajectory. Lesotho and Nicaragua's top enterprises are foreign-owned and part of big Asian supplier networks. These corporations adopt business strategies in which high-value upstream and downstream operations are performed in their Asian headquarters, with limited links or technological spillovers to local suppliers. Neither nation has upgraded much. Locally held enterprises play major roles in Bangladesh, Sri Lanka, and Turkey, with direct links to global customers who have upgraded local operations.

The public and private sectors must commit to industry growth to upgrade to ODM and OBM. Turkey is the only nation in our sample to make large breakthroughs in ODM and OBM. Strong industry groups and government organizations collaborated to boost Turkey's fashion and design competitiveness. Turkey's major integrated enterprises' full-package skills promote tight partnerships with global merchants that are eager to help upgrade Turkey's design and brand services. Sri Lanka's government and corporate sector established a 5-year strategy to enhance the industry, focusing on leveraging their tight relationships with global customers to build design and brand competencies. Sri Lankan enterprises have offices in important locations to cooperate with product development and design teams.

## 8. Conclusion

One of the businesses that have seen the greatest degree of globalization in our day is the clothing industry. It is responsible for the employment of millions of people all around the globe, particularly in nations with low incomes. The ability of developing nations to join the value chain may be attributed to a number of crucial factors, including the availability of low-cost labor, advantageous trade agreements, and closeness to end markets. Workforce development programs receive little attention, despite the fact that the companies that dominate this value chain have strict requirements for their suppliers. Supervisors who can't instruct manufacturing workers often do so. Vocational schools don't provide courses that meet industry demands. Many firms feel expatriates are more efficient than native personnel. The influence of global purchasers to improve working conditions and moves in more mature suppliers to professionalize the clothing workforce imply that developing nations are coming closer to adopting more effective and meaningful workforce development procedures. This is because global buyers are working to improve working conditions. It devised a comprehensive industrial strategy with the goal of promoting industrialization through fostering the growth of the manufacturing industry, with textile and garment production being among the highest priority sectors. It has utilized governmental levers to give assistance to exporters without opening up the domestic market to international goods and FDI enterprises, allowing it instead to be dominated by indigenous businesses. The government has implemented a number of buyer attraction strategies in addition to actively seeking foreign direct investment from key garment manufacturing nations. One of the most important tools for luring in new investment is the creation of serviced industrial parks that provide specific advantages to businesses who export their products. It has supported integration between the production of textiles and clothing as well as the cotton industry in order to achieve the goal of creating a local value chain that is integrated. In addition to facilitating knowledge linkages between the industry and higher education institutions, it has created sector-focused institutions with a primary focus on building technological capability and capabilities in terms of skills, with managers, technicians, and workers as its primary targets. This research will be of significant value for specialists in choosing an acceptable and rigorous technique for sustainability evaluation in the textile sector. In a similar vein, due to the one-of-a-kind nature of the textile and apparel industry, it is essential for the researcher to carry out research that is both more universal and comprehensive on the topic of sustainability in this sector, and then use the findings to outline the directions in which they intend to take their future research. The evaluation levels, limits, source, and weight of indicators that are discussed in this research may be used as a checklist, and they cover the majority of the characteristics of the textile and clothing business. The prioritizing of source and weight of indication will aid the investors of textile apparel and industry in making the trade-off between multiple performances and measures. Furthermore, the assessment of the reviewed studies showed that the economy is the most researched and enhanced measurement in the garment industry although both social and economic aspects still demonstrate some struggles in their quantification because of a lack of applicable and measurable indicators. Therefore, we need to improve the relationship between apparel value chains and SEDs and then the global organization of the apparel design industry. The research refers to an overall sort of assessment of the textile and apparel sector and may be used to evaluate the textile industries of both developed and developing countries to determine how well they perform in terms of sustainability [53].

## Figures and Tables

**Figure 1:** Sustainable growth in each country.

**Figure 2:** Principles of achieving sustainability.

**Figure 3:** Apparel global value chain.

**Figure 4:** Apparel global value chain's curve of value-added stages.

**Figure 5:** Economic upgrading for the apparel industry.

**Figure 6:** Sustainable development of the apparel industry.

**Table 1:** Employment in the apparel industry in a few countries.

Regions	Employment	The ratio of the overall manufacturing employment (percent)	Year
Nicaragua	80,510	27	2006
Cambodia	2,52,000	39	2005
Turkey	5,01,000	15	2009
China	19,100,000	20	2004
India	463,320	7	2001
Sri Lanka	2,71,000	21	2008
Madagascar	88,000	44	2001
Mauritius	76,964	65	2001
Morocco	1,76,895	19	2002
Mexico	4,610,000	11	2005
Pakistan	2,310,000	44	2001
Bangladesh	2,810,000	—	2008
Romania	403,390	24	2002
Guatemala	104,465	22	2005
Lesotho	40,363	—	2005

## Data Availability

The data used to support the findings of this study are available from the corresponding author upon request.
